This article has been retracted.

# Effect of Integrated Psychobehavioral Care on Emotional-Behavioral Responses, Cognitive Changes in Outpatients with Schizophrenia Followed Up: Based on a Prospective Randomized Controlled Study

**DOI:** 10.1155/2022/1862396

**Published:** 2022-06-16

**Authors:** Yao Yao, Yali Xu, Hongyan Guo, Kunxiu Han, Zhuo Dai

**Affiliations:** ^1^Department of Outpatient, Nanjing Jinling Hospital, Nanjing University School of Medicine, Nanjing, 210002 Jiangsu Province, China; ^2^The Sixth Stationed Outpatient Department, Nanjing Jinling Hospital, Nanjing University School of Medicine, Nanjing, 210002 Jiangsu Province, China; ^3^Department of Health Medicine, Nanjing Jinling Hospital, Nanjing University School of Medicine, Nanjing, 210002 Jiangsu Province, China; ^4^Department of Invasive Technology, Nanjing Jinling Hospital, Nanjing University School of Medicine, Nanjing, 210002 Jiangsu Province, China; ^5^Department of Burn and Plastic Surgery, Nanjing Jinling Hospital, Nanjing University School of Medicine, Nanjing, 210002 Jiangsu Province, China

## Abstract

**Background:**

In recent years, influenced by the continuous improvement and development of the medical service model and the increasing demands of modern people for the quality of clinical care, the clinical treatment of schizophrenic groups has also received widespread attention and importance from all sectors of society. Psychobehavioral care is administered to patients during active antipsychotic treatment, which can maximize the patient's cooperation with clinical work and thus play an auxiliary role in treatment.

**Aims:**

To investigate the impact of emotional-behavioral responses, cognitive changes in outpatient follow-up of schizophrenic patients with integrated psychobehavioral care.

**Materials and Methods:**

One hundred cases of schizophrenia patients with outpatient follow-up in our hospital from March 2017 to March 2019 were selected as prospective study subjects and divided into a comparison group and an observation group of 50 cases each according to a random number table. Among them, the comparison group implemented conventional psychobehavioral care, and the observation group implemented integrated psychobehavioral care. The differences in compliance behavior, negative emotions, cognitive behavioral changes, and pain scores before and after care of schizophrenia patients in the outpatient follow-up were compared between the two groups.

**Results:**

After care, the compliance behavior, negative emotions, cognitive behavioral changes, and pain scores of schizophrenia patients in both groups with outpatient follow-up were significantly improved and significantly higher in the observation group than in the comparison group, and statistics showed that this difference was statistically significant (*P* < 0.05).

**Conclusion:**

Integrated psychobehavioral care combined with conventional psychobehavioral care can effectively enhance the compliance behavior of outpatient follow-up schizophrenia patients, improve the negative emotions and pain of patients, and facilitate the active treatment of patients to improve their prognosis. It has some reference value for outpatient follow-up schizophrenia patient care.

## 1. Introduction

Schizophrenia affects patients' emotions, behavior, thinking, and perception [1]. Schizophrenia is a recurrent illness with high relapse and disability rates, often accompanied by social skill deficits and high rates of perpetration and accidents in schizophrenic patients, which seriously interfere with the life and safety of the community [2]. Due to the special national conditions in China, the restoration of patients' social functions and relapse prevention are of great importance to their family impact, and although various antipsychotic drugs can effectively control their psychiatric symptoms, they cannot help their impaired social functions and psychiatric disability, which seriously affects patients' quality of life [3]. Prevention of schizophrenia relapse and improvement of the quality of life of schizophrenia patients are of increasing concern to the majority of psychiatric medical practitioners and patients' families [4]. Striving for early and standardized antipsychotic treatment plays an important role in improving the aforementioned symptoms in schizophrenia patients, but the expected results are often not easily achieved by providing patients with pharmacological interventions alone due to a variety of factors [5]. In recent years, influenced by the continuous improvement and development of the medical service model and the increasing requirements for the quality of clinical care put forward by modern people, the clinical treatment of schizophrenia groups has also received wide attention and importance from all walks of life [6]. Therefore, this study provides some reference basis for the clinical care of schizophrenia patients in outpatient follow-up by examining the effects of emotional-behavioral responses and cognitive changes in schizophrenia patients using integrated psychobehavioral care, which is reported below.

## 2. Material and Methods

### 2.1. Research Object

In this study, the regression of solid tumors was calculated according to the sample size of the cross-sectional survey: *n* = *t*_*a*_^2^*PQ*/*d*^2^, where *n* was the sample size, *P* was the incidence of schizophrenia, *Q* = 1 − *P*, and *d* was the allowable error. *a* = 0.05; ta = 1.96. The minimum sample size brought into the formula is 95 cases. In this study, 100 cases of outpatient follow-up schizophrenia patients were actually included as study subjects. Patients with outpatient follow-up schizophrenia who met the inclusion criteria were numbered according to a random number table and randomized into 50 cases each in the control and observation groups using the random number table of the third edition of Medical Statistics [7]. No characteristic information about the patients was extracted or accessed during the study, and therefore, no ethical review or waiver of authorization or exemption from informed consent was required.

### 2.2. Exclusion Criteria

Inclusion criteria are as follows: (1) selected outpatient follow-up schizophrenia patients were in accordance with the Guidelines for the Treatment of Schizophrenia [8] and met the Chinese Classification and Diagnostic Criteria of Mental Disorders, 3rd edition (CCMD-3) diagnostic criteria for schizophrenia; (2) Brief Psychiatric Rating Scale (BPRS) score ≥ 35, first onset and duration of illness ≤2 years, no previous systematic antipsychotic treatment, and age 16 to 45 years; and (3) patients with ≥6 years of education and at least one guardian who had supervised the patient for 1 year and obtained informed consent from the guardian. Exclusion criteria are as follows: (1) comorbidities of other heavy mental illnesses, mental retardation, dementia and severe cognitive dysfunction, unwillingness, or inability to cooperate continuously for a specified period of time for various reasons; (2) those who have used psychosis-related drugs in the past 3 months. Selected patients with severe heart, liver, kidney, and other physical diseases and inability to cooperate due to special family and personal; and (3) patients with intellectual disabilities and alcohol and drug dependence.

### 2.3. Methods

#### 2.3.1. Conventional Psychobehavioral Care

Patients are managed in the traditional family care model of closed care for the treatment of mental illness, which reduces the patient's contact with the outside world and prevents the patient from aggravating his or her condition due to the stimulation of the outside environment. Family members are responsible for specific care management, such as medication, diet, and observation of symptoms, and doctors adjust the treatment plan according to the condition at follow-up visits.

#### 2.3.2. Integrated Psychobehavioral Care

Establish outpatient follow-up files, send doctors and senior nurses into the community, and follow up and care for patients within 3 months after discharge every 15 d. Follow up by phone for those who cannot enter the community and once a month for 6 months after discharge.

*(1) Psychological Care*. The psychological intervention was implemented by 2 deputy chief psychiatric nurses and 5 competent nurses, and its contents included the following: (1) health education: including the following 6 topics: understanding schizophrenia and psychiatric symptoms; knowledge about schizophrenia medication; course, outcome, and relapse of schizophrenia; family care of schizophrenia patients; rehabilitation of schizophrenia patients; and marriage of psychiatric patients. The following are some of the topics covered in this course. (2) Social skills training: including the following six topics: mutual self-introduction and name explanation and back-to-back drawing games; how to find help; conversation process skills training (such as body distance training, eye contact, and posture skills training); learning how to deal with people; how to cooperate with others; and through role-playing to show the conflict problems in daily life with people, learn to analyze and solve the problems that arise in the social process. (3) Vocational rehabilitation training: including rehabilitation training (self-service initiation lack of training, recreation) and problem-solving skills training. (4) Group cognitive psychotherapy: according to the theory of cognitive therapy, the patient's distorted irrational thinking and behavior are replaced by rational thinking, adjusting his interpersonal relationships, enhancing his compliance with medication, and improving his self-confidence. Based on the patient's personality characteristics and the environment and home care they live in, a community management system is established to assess care problems and develop a complete community care plan to provide comprehensive psychiatric rehabilitation training for patients. The postintervention situation is analyzed and evaluated monthly, problems are raised and treatment plans and nursing interventions are revised accordingly, and learning about mental health and the physical and psychological characteristics of the period is conducted from time to time in the form of group talks, brochures, and training courses to raise the awareness of chaperones and patients about schizophrenia, so that chaperones know how to properly store medications and treat patients and how to care for.

*(2) Behavioral Care*. (1) Teach general knowledge about schizophrenia; (2) assess the different degrees of behavioral disorders and give targeted adjustment and correction; (3) help patients identify abnormal behaviors and recognize them; (4) correct bad habits; (5) train patients' interpersonal skills; (6) carry out cultural and sports activities according to patients' interests or play intelligent games according to patients' tendency of mental decline; and (7) encourage patients to freely associate with each other, so that they can help each other and find their own value or emotional experience.

### 2.4. Observation Indicators

Patients' compliance behaviors, negative emotions, cognitive behavioral changes, and pain scores were assessed before and after care. The higher the score, the better the compliance behavior of schizophrenia patients in outpatient follow-up. A compliance questionnaire was used to measure the compliance behavior of patients in both groups after 6 months of nursing intervention. The questionnaire on medical compliance behavior mainly investigates 7 dimensions: regular physical examination, taking medicine on time, regular testing, outpatient follow-up, maintaining stable emotions, doing things within one's ability and participating in social activities, and doing what they can and participating in social activities. (1) Self-efficacy score: a total of 10 items, each of which is 1-4 points; the higher the score, the better the patient's self-efficacy. (2) Negative mood score was evaluated based on the Brief State of Mind Scale (BPOMS), including four items: anxiety, depression, fatigue and sleepiness, and anger, each with 0-7 points; the higher the score the greater the negative mood. (3) Cognitive-behavioral score: including two items of patients' cognitive degree and behavioral change for outpatient follow-up, each item has 15 subitems, each item has a total of 30 points; the higher the score, the worse the cognitive behavior. (4) Pain score: visual analogue scale (VAS) score was used, with a total of 10 points, and the higher the score, the more severe the pain. It was measured before and after nursing care. (5) Brief Psychiatric Symptom Rating Scale (BPRS): total score of 18-126, reflecting the severity of the disease; the higher the total score, the more severe the disease, and the change in the total score before and after treatment reflects the efficacy of the treatment; the greater the difference, the better the efficacy. The general study group standard can be set at 35 points. The individual scores 0-7 reflect the distribution of symptoms and the severity of target symptoms. The change before and after treatment can reflect the change of target symptoms of treatment. Because BPRS is a graded scale, it can reflect the efficacy of treatment in a more detailed way. The above rating scales have good reliability and validity, and the joint examination consistency *r* = 0.787 when applied to patients with schizophrenia. The consistency of single-item ratings of repeated examinations = 0.77, except for anxiety, nervousness, and peculiar behavior posture, *P* was less than 0.05. The positive-negative agreement rate between the scale ratings of each single symptom and clinical records, Kappa = 0.37. All were significant except for one item of suspicion. The correlation between its total score and the grade of clinical severity = 0.84; the correlation with the judgment of clinical efficacy *r* = 0.6.

### 2.5. Statistical Analysis

All statistical data in this study were entered into Excel software by the first author and the corresponding author, respectively, and the statistical processing software was SPSS25.0 for calculation. Repeated measure analysis of variance between groups was used to measure the measurement expressed as mean ± standard deviation (*X* ± *S*). material. Count data expressed as a percentage (%) were tested by *χ*^2^. Univariate and Logistic multivariate regression analysis was used to compare the influencing factors, and the risk factors with significant differences were screened. Univariate and logistic multivariate regression analysis was used to compare the influencing factors, and the risk factors with obvious differences were screened. The statistical significance was *P* < 0.05.

## 3. Results

### 3.1. Analysis of General Data

There was no statistically significant difference between the two groups of outpatient follow-up schizophrenia patients in terms of general data such as gender, mean age, duration of illness, and education level by *t*-test and chi-square test (*P* > 0.05) (see Table 1).

### 3.2. Comparison of Medical Compliance Behavior Scores

Before nursing, there was no significant difference in the scores of compliance behavior between the two groups of patients with schizophrenia during outpatient follow-up (*P* > 0.05). After nursing, the two groups of patients with schizophrenia were followed up in the outpatient clinic for their psychological behavior scores, exercise status scores, drug taking scores, balanced diet scores, regular physical examinations, regular tests, outpatient follow-up visits, maintaining stable emotions, doing things within their ability, and participating in social activities. The number of people who took medicine on time was significantly improved, and the observation group's compliance behavior score was significantly higher than that of the control group, and statistics showed that the difference was statistically significant (*P* < 0.05) (see Figures 1 and 2).

### 3.3. Comparison of Negative Mood Scores

Before care, there was no statistically significant difference in the negative mood scores between the two groups of schizophrenia patients at the outpatient follow-up (*P* > 0.05). After care, the anxiety, depression, fatigue, and anger of schizophrenia patients at the outpatient follow-up in both groups improved significantly, and the negative mood scores of the observation group were significantly lower than those of the comparison group, which was statistically significant (*P* < 0.05) (see Figure 3).

### 3.4. Comparison of Cognitive-Behavioral Changes and Pain Scores

The cognitive behavioral changes and pain scores of schizophrenia patients at outpatient follow-up in both groups improved significantly after care and were significantly less in the observation group than in the comparison group, with a statistically significant difference (*P* < 0.05) (see Figure 4).

### 3.5. Comparison of BPRS Scores

Before care, there was no statistically significant difference in BPRS scores between the two groups of outpatient follow-up schizophrenia patients (*P* > 0.05). After care, the anxiety and depression, lack of energy, dysfunctional thinking, activation, and hostile suspicion of the schizophrenic patients at the outpatient follow-up in both groups improved significantly, and the negative mood scores in the observation group were significantly lower than those in the comparison group, which was statistically significant (*P* < 0.05) (see Figure 5).

## 4. Discussion

Schizophrenia is a serious mental illness that seriously endangers human health, with a prolonged course and high relapse and disability rates, causing heavy family and social burdens and seriously affecting patients' quality of life [9]. Various types of antipsychotic drugs currently play a great role in relieving schizophrenic psychiatric symptoms in the acute phase, but they are still unsatisfactory in preventing relapse and improving social functioning [10]. Therefore, most schizophrenic patients who have returned to society, including those who respond well to medication, are likely to relapse and be hospitalized again due to their deficits in social functioning even when they adhere to medication [11]. Active and effective psychosocial interventions for patients with schizophrenia have been reported to delay or reduce the degree of impaired social functioning and psychiatric disability, allowing them to return to society and maintain a high quality of life [12]. At present, most schizophrenia patients in China are hospitalized under closed management, resulting in a restricted range of activities, for which patients often feel dissatisfied with the hospitalization environment, and some of them may be hostile to medical and nursing staff, uncooperative with treatment and care, refusing to communicate with their patients and refusing to participate in various activities organized by the hospital [13]. In order to reduce or eliminate these phenomena, relevant studies have found that patients' cognitive function can be improved more significantly than conventional care after psychobehavioral interventions. In the present study, the authors were largely in agreement with this view [14]. Psychobehavioral interventions can reduce the psychological burden of patients through cognitive interventions, emotional reassurance, and behavioral guidance, guide patients to treat their condition correctly, and allow them to exercise all aspects of their abilities in an orderly manner according to the rehabilitation plan [15]. Compared with conventional care, this model is more in line with the person-centered concept advocated by modern nursing and more effective in promoting the recovery of patients' conditions [16]. We provided targeted psychological interventions for patients in the observation group to train their interpersonal and social adaptation skills. During the training process, patients were provided with various learning knowledge, exchanged their experiences of the disease with each other, discussed the difficulties encountered in real life, and provided each other with opportunities for support and understanding so that they could face reality, eliminate negative cognitions, enhance their self-confidence and self-esteem, and improve their psychological stress capacity, thus laying the foundation for improving patients' social functioning [17].

This study investigated the effects of integrated psychobehavioral care on emotional-behavioral responses and cognitive changes in outpatients with schizophrenia at the outpatient follow-up. This difference was statistically significant. It is suggested that the integrated psychobehavioral care can effectively enhance the compliance behavior of schizophrenia patients in the outpatient follow-up, which is conducive to the active treatment and prognosis of patients. In this study, we found that outpatient follow-up schizophrenia patients rarely communicate with medical staff actively at first but communicate with other patients through social software, deliberately concealing symptoms and psychological needs to reduce the burden on family members but lacking active guidance from nurses, and communication solely among patients may lead to adverse consequences [18]. The psychological burden of patients was greatly reduced by making them talk and listen to each other through correcting misperceptions, emotional support, and care of maladaptive behavioral habits, such as encouraging patients to get out of bed and exercise appropriately, listen to soft music, muscle relaxation, and deep breathing exercises [19].

In this study, the anxiety, depression, fatigue, and anger of schizophrenia patients in both outpatient follow-up groups were significantly improved, and the negative mood scores of the observation group were significantly lower than those of the comparison group, and statistics showed that this difference was statistically significant. The cognitive behavioral changes and pain scores of schizophrenia patients in both outpatient follow-up groups were significantly improved, and the observation group was significantly less than the comparison group, and this difference was statistically significant in comparison. It is suggested that integrated psychobehavioral care combined with conventional psychobehavioral care can effectively enhance outpatient follow-up schizophrenia patients to improve patients' negative emotions and pain, which is conducive to active treatment of patients to improve their prognosis. Anxiety and depression are the two most common negative emotions in patients; anxiety is an irritability caused by excessive fear for the safety of life and future fate of loved ones or ones [20]. Depression is a negative emotion such as pessimism, sadness, and despair. Integrated psychobehavioral care is an advanced care model that was aimed at improving patients' lives after discharge by implementing effective health education and increasing their awareness of outpatient follow-up [21]. Nursing staff instructed patients to eat a reasonable diet and prohibited them from consuming foods high in uric acid to reduce the recurrence rate of calcium-containing stones.

The results of this study showed that the use of home follow-up and psychological care interventions for patients with schizophrenia significantly improved patients' compliance behavior and quality of life, and the relapse rate decreased significantly. This suggests that follow-up and psychological care interventions are effective primary care tools for patients after discharge from the hospital. In the process of giving patient care, patients and patients' families were empowered to recognize the disease and fully understand the importance of adhering to medication in compliance with medical advice for treatment [22]. The patient's family members, under the guidance of the medical staff, maintain a good relationship with the patient, actively communicate with the patient, and give the patient emotional support so that the patient feels the warmth of the family and enhances the confidence to overcome the disease [23]. Giving corresponding psychological guidance according to different patients' different psychological states can effectively improve their mental health problems such as anxiety, depression, terror, hostility, and interpersonal sensitivity. A large number of clinical practices have shown that administering psychobehavioral care to patients during active antipsychotic treatment can maximize patients' cooperation with clinical work, which in turn can be an adjunct to treatment [24]. Related studies have found that after psychobehavioral interventions, patients' cognitive function can be improved more significantly than with conventional care [25]. In the present study, the authors were largely in agreement with this. Psychobehavioral intervention can reduce patients' psychological burden through cognitive intervention, emotional reassurance, and behavioral guidance, guide patients to treat their condition correctly, and allow them to exercise all aspects of their abilities in an orderly manner according to the rehabilitation plan. Compared with conventional care, this model is more in line with the person-centered concept advocated by modern nursing and is more effective in promoting the recovery of patients' conditions .

The results of this study showed that the use of integrated psychobehavioral care in combination with conventional psychobehavioral care intervention for patients with schizophrenia significantly improved patient compliance and quality of life, and the relapse rate decreased significantly. This suggests that the combination of psychobehavioral care and psychobehavioral care interventions is an effective primary care tool for patients after discharge. In the process of giving patient care, patients and their families are empowered to be aware of the disease and fully understand the importance of adhering to medication as prescribed for treatment [26–29]. Under the guidance of the medical staff, the patient's family members maintain a good relationship with the patient, actively communicate with the patient, and give the patient emotional support, so that the patient feels the warmth of the family and has increased confidence in overcoming the disease [30]. Giving appropriate psychological guidance to different patients according to their different psychological states can effectively improve their mental health problems such as anxiety, depression, terror, hostility, and interpersonal sensitivity [31]. Outpatient follow-up files and rational treatment and personalised community care plans are established to implement interventions in all aspects of the patient's life environment, cognitive education, and patient behavioral situations [32–35]. During the training process, patients are provided with a variety of learning knowledge, share their experiences of the disease with each other, discuss the difficulties they encounter in real life, and provide each other with opportunities for support and understanding so that they can face reality, eliminate negative cognitions, enhance their self-confidence and self-esteem, and improve their psychological stress capacity, thus laying the foundation for improving their social functioning [36–39]. As patients' life skills and social skills improve, they will actively participate in group activities, making their inpatient life more enriching and improving their quality of life. The establishment of an outpatient follow-up file combined with community nursing interventions and the designation of professionals will enable a full understanding of the patient's situation, timely modification of the treatment plan, and the development of individualised interventions [40]. Comprehensive psychiatric rehabilitation training for patients can effectively improve treatment compliance, facilitate the recovery of adolescent schizophrenia patients, improve social readjustment and quality of life, and reduce the burden on families and society and is worth promoting in clinical practice. The advantages of this study are as follows: integrated psychobehavioral care significantly improved patient compliance behavior and quality of life, and the recurrence rate was significantly reduced. It is suggested that integrated psychobehavioral care is an effective main nursing method for patients after discharge. In the process of giving patient care, enhance the cognitive ability of patients and their family members on the disease, and fully understand the importance of adhering to the doctor's advice to take medicine for treatment. Family members of patients maintain a good relationship with patients, actively communicate with patients, and provide emotional support to patients, so that patients feel the warmth of their families and enhance their confidence in overcoming the disease.

This study has some innovations and some limitations. First, the patients with schizophrenia included in this study were not cared for according to specific categories, and the selected patients with schizophrenia in outpatient follow-up were all from our hospital's outpatient follow-up schizophrenia patients, so the selection of patients included to exclude outpatient follow-up schizophrenia was somewhat subjective, and the study results may not be representative or biased. Psychobehavioral interventions have more limitations in practice, such as lack of understanding of patients and their family situations, economic conditions, uneven allocation of medical resources, and many other factors that can affect patients' emotions, which could not be assessed comprehensively and systematically in this study.

In conclusion, integrated psychobehavioral care combined with conventional psychobehavioral care is effective in enhancing the compliance behavior of schizophrenia patients in outpatient follow-up, improving patients' negative emotions and pain, and contributing to positive patient treatment and prognosis. It has some reference value for outpatient follow-up schizophrenia patient care.

## Figures and Tables

**Figure 1:** Comparison of the medical compliance behavior of the two groups of patients (the count data of the medical compliance behavior of the follow-up patients are represented by integers, and the chi-square test was used to find that after the nursing, the two groups of patients had regular physical examinations, regular tests, and outpatient follow-up visits, maintained stable emotions, and did their best. The number of people participating in social activities and taking medicines on time was significantly improved, and the observation group's compliance score was significantly higher than that of the control group, and the difference was statistically significant (*P* < 0.05)).

**Figure 2:** Comparison of the scores of medical compliance behavior between the two groups (the measurement data in this study were entered in Epidata and expressed as mean ± standard deviation (*x* ± *S*), and SPSS 25.0 was used for statistical processing of the data, and the data needed to be entered into the computer by a personnel. The database was checked and revised by a second person to ensure the completeness and accuracy of the data. Using independent samples *t*-test, it was found that after care compared to before care, the psychological behavior scores (a), motor condition scores (b), medication taking scores (c), and balanced diet scores (d) of schizophrenia patients in both outpatient follow-up groups were significantly improved, and the compliance behavior scores of the observation group were significantly higher than those of the control group, which statistically showed a statistically significant difference (*P* < 0.05)).

**Figure 3:** Comparison of negative emotion scores between the two groups of patients (the measurement data in this study were entered into Epidata, expressed as mean ± standard deviation (*x* ± *S*), and SPSS 25.0 was used for statistical processing of the data, and the data are needed to be entered into a computer database by a second person to check and modify to ensure the completeness and accuracy of the data. Using independent samples *t*-test, it was found that the anxiety score (a) and depression score (b) of the two groups of outpatient follow-up schizophrenia patients after nursing were compared with those before nursing. The score of fatigue and distress (c) and the score of anger (d) were significantly improved, and the negative emotion score of the observation group was significantly lower than that of the control group, and the difference was statistically significant (*P* < 0.05)).

**Figure 4:** Comparison of cognitive behavioral changes and pain scores in the two groups (the second person checked and revised to ensure the completeness and accuracy of the data. Using an independent sample *t*-test, it was found that the cognitive level of the schizophrenia patients in the outpatient follow-up in the two groups after nursing was compared with that before nursing (a); behavior changes (b), pain score (c), and self-efficacy (d) were significantly improved, and the observation group was significantly less than the control group, and the difference was statistically significant (*P* < 0.05)).

**Figure 5:** Comparison of the BPRS scores of the two groups of patients (the BPRS scores included in this study were measurement data, expressed as the mean ± standard deviation (*X* ± *S*), and were checked and corrected by a second person to ensure the integrity and accuracy of the data. Independent sample *t*-test found that patients with schizophrenia have anxiety and depression (a), lack of energy (b), thinking disorder (c), activation (d), hostile suspicion (d), and the hostile suspicion (e) significantly improved, and the negative emotion score of the observation group was significantly lower than that of the control group; the difference was statistically significant (*P* < 0.05)).

**Table 1:** Comparison of general information between two groups of patients [*n*, ($\bar{x}\pm s$)].

Group	Gender (male/female)	Average age (years)	Duration of illness (months)	Education level	
				College and above	High school and below
Comparison group (50)	32/18	26.31 ± 3.51	12.98 ± 4.52	24	26
Observation group (50)	31/19	26.30 ± 3.52	12.75 ± 4.02	22	28
*χ* ^2^ */t*	0.043	0.032	0.269	0.161	
*P*	0.836	0.975	0.789	0.688	

## Data Availability

No data were used to support this study.
